The article "Evaluation of Physical Education Teaching Effect Based on Action Skill Recognition" was published in 2022. Journal: Comput Intell Neurosci.

# Evaluation of Physical Education Teaching Effect Based on Action Skill Recognition

**DOI:** 10.1155/2022/9489704

**Published:** 2022-05-31

**Authors:** Xia Ding, Wei Peng, Xiaoling Yi

**Affiliations:** ^1^School of Teacher Development, Chongqing University of Education, Chongqing 400065, China; ^2^Physical Education Teaching and Research Section, Chongqing No. 2 Foreign Language School, Chongqing 400065, China; ^3^Student Development Centre, Chongqing Long Men Hao Vocational School, Chongqing 400000, China

## Abstract

In order to improve the effect of physical education teaching in modern colleges and universities, this paper combines the movement skill recognition algorithm to construct a physical education effect evaluation system and studies the multispectral image reproduction system in practical application. Moreover, this paper gives a detailed description of more advanced functional modules in the system, such as spectral acquisition, spectral reflectance reconstruction, and spectral color correction. In addition, this paper focuses on the algorithm design of the color appearance matching module. By adding the “color appearance transformation” on the source side and the “color appearance inversion” on the reproduction side, the source image and the reproduced image can achieve color appearance matching in the observation condition-independent space. The simulation experiment verifies that the physical education effect evaluation system based on action skill recognition meets the actual needs of physical education and has a good role in promoting the recognition of physical skills and the improvement of physical education effect.

## 1. Introduction

In the process of physical education teaching innovation, teachers should learn more ways to develop students' creativity, create a good educational situation for students, enable students to put forward their own views on the corresponding issues relatively independently, and ensure a good atmosphere for physical education teaching. In this way, students' creative awareness will be improved, and they will be able to carry out sports learning more flexibly. A successful physical education class is composed of many elements, such as experienced physical education teaching, students with strong curiosity, scientific teaching mode, and sports equipment. These physical education classroom elements are interrelated, but sometimes they are opposite to each other to a certain extent. The change of each element may lead to the change of another element, and the quality of physical education teaching may also be affected. In this case, in order to make the innovation and cultivation of physical education successful, it is necessary to consider from a global perspective and seriously consider the connections between different elements. Only in this way can sports innovation teaching be carried out better and better results can be achieved.

Physical education space is not a purely material concept but the real life and the living conditions shared by teachers and students in the process of physical education. It is a humanistic structure full of life and cultural significance. Moreover, the physical education space contains political power, social relations, cultural dependence, psychological activities and other material, spiritual factors, and social factors. Materiality is the space that can be directly observed, spirituality is the space constructed by language, and sociality is the relational space between teachers and students, teaching and learning, and teaching and the environment. The extraordinary thing about physical education teaching space is that it is not a space for simple language construction but a space for artistic reproduction of body language—a practical space for showing sports technology. Moreover, it is a spatial concept that organically integrates materiality, spirituality, and sociality through the practice of physical education, so it also has more vitality and cultural significance.

The practical activities of physical education teachers and students and their discourse tendencies are first placed in the space, because the elements of the whole process of physical education, including physical education teachers, students, physical education concepts, physical education methods, and physical education effects, are presented in the space, in a specific space. “Space is the mediator of social action and actively affects social action. Space is the raw material of social process and also the product of social process”. In the special environment of physical education teaching, spatial behavior is the result of the mutual penetration and interaction of physical education teacher's ability, students' quality, spatial situation, and social culture. Physical education teachers' grasp of space theory and its value directly affects the effect of physical education teaching. Every demonstration action of physical education teachers is a spatial art reproduction of body language. However, in reality, physical education teachers are constrained by the cultural environment, the background of the times, cognitive ability, and living customs, and they do not realize the priority of space in physical education teaching. In teaching practice, the measure of time conceals the priority of space. The weak concept of space does not only exist in physical education teachers. Students ignore the self-constructed space in the practice of physical activities and pursue the so-called autonomy. The basis of students' autonomous sports practice is the mastery of individual motor skills. Needless to say, it takes time for students to master motor skills.

This paper combines the movement skill recognition algorithm to construct the physical education effect evaluation system and promote the progress and development of the modern physical education reform.

## 2. Related Work

This study proposes a new image stitching algorithm based on contour features. In the feature extraction stage, the convolution map is enhanced and the region growth method is used for auxiliary correction, which can improve the contour extraction effect; in the aspect of feature representation, the shape signature is used instead of the chain code to describe the contour, which improves the calculation speed and reduces the cost of effects of noise interference and lens distortion [1]. Aiming at the continuous stitching of sequence images with translation, rotation, and scaling transformation, a stitching algorithm combining the registration algorithm based on regional features and the registration algorithm based on gray cross-correlation is proposed. The algorithm extracts regions with an iterative threshold segmentation algorithm, uses region features for registration, establishes an initial pair of regions with the same name, then uses the centroid points of the pair of regions with the same name as feature points, and selects the cross-correlation criterion as a metric based on the grayscale information of the image. Finally, the accurate transformation relationship between images is obtained, and the stitching of sequence images is realized [2]. An image feature matching algorithm based on Laplacian matrix is proposed. First, we construct the Laplacian matrix of the feature point sets of the two images, respectively, perform singular value decomposition (SVD) on the two matrices, and then use the decomposition result to construct a relationship matrix that reflects the matching degree between the feature points to achieve the feature point which matches the two images [3]. The traditional template matching algorithm is studied and analyzed, and a new fast template matching algorithm based on projection is proposed. The two-dimensional image is one dimensionally projected, and the one-dimensional projection value is further differentially quantized to obtain a set of character strings consisting of 0 and 1 numbers that describe the image and the template. The KMP fast character matching algorithm is introduced to directly compare the image and template [4]. A two-stage correlation matching improvement method is proposed, and a fast hierarchical pyramid matching algorithm is constructed [5]. Based on the principle of template matching, a new automatic color image stitching method is proposed [6]. For two-color images with overlapping areas, the method first uses the image feature information to automatically find a small template image from the overlapping area of one image and then searches in the overlapping area of the other image according to the maximum similarity criterion. When the best image registration point is found, the final data fusion operation is performed on the overlapping area of the two images by using the smoothing factor, which can realize the fast and automatic stitching of color images [7]. Two similarity measurement methods, sequential similarity detection (SSDA) and normalized product correlation, are used to establish the similarity measurement value between the template image and the input image and then used the simulated annealing algorithm to randomly search for the optimal solution quickly and accurately—best match. At the same time, on the other hand, stitching in the frequency domain and phase has become one of the new research hotspots. The fact that its unique stability and the characteristics that it have are not easily affected by the change of image grayscale errors has attracted the attention of relevant researchers. A lot of research work has been done in this area and many attentions have been made to [8]. Using a tightly supported vector wavelet with orthogonality and symmetry, the two images were mosaicked and spliced. Because the wavelet transform has the property of a band-pass filter, the wavelet transform components at different scales actually occupy a certain bandwidth and scale. The larger the value, the higher the frequency of the component; so the bandwidth of each wavelet component is not large, the two images to be spliced are first decomposed into wavelet components of different frequencies according to the method of wavelet decomposition, then in different scales under different stitching widths, the two images are first stitched together according to the wavelet components of different scales, and then, the restoration program is used to restore the entire image [9]. The research expands the application scope of the image registration method based on Fourier–Mellin transform from two aspects. The first is the stitching of panoramic images, and the other extension is the matching of image curves [10]. The image curves are converted into binary images, and then, the Fourier–Mellin transform is applied to register these binary images, so as to match the two curves [11].

The grayscale-based segmentation method is intuitive and easy to operate and is widely used in practice. However, due to the influence of image grayscale distortion and various environmental factors, it is easy to cause mis-segmentation. For this problem, many scholars have given great energy and designed various algorithms to solve it [12]. However, due to the influence of various factors, the grayscale image segmentation method still cannot completely solve the problem of incorrect segmentation and excessive segmentation error. Analyzing the reasons for the oversegmentation of the watershed algorithm, simplifying the grayscale transformation, and using the influence of different structural elements of mathematical morphology on the distance transformation, an improved algorithm combining the watershed and Livewire is proposed, which can reduce the oversegmentation effect and make the calculation more efficient [13]. Aiming at the two defects of the watershed segmentation algorithm, time consuming and oversegmentation, a multiresolution-based watershed image segmentation algorithm is studied. This algorithm performs watershed segmentation on low-resolution images and improves the speed of segmentation [14]. When returning from a low-resolution image to a high-resolution image, a merging function based on edge information is used to avoid the loss of edge information and ensure the accuracy of segmentation [15]. A noise suppression method based on gradient images is designed, which can suppress the influence of Gaussian noise on gradient images and effectively avoid the problem of over-segmentation [16].

## 3. Action Recognition Algorithms

The multispectral image reproduction process in practical application is shown in Figure 1. Among them, the spectral image input device and the illumination light detection device are used for spectrum acquisition to obtain the reflection spectrum and the illumination light spectrum of the scene object and to provide a data source for computer processing. Computers are used for operations such as spectral reflectance reconstruction. When the spectral reproduction is remote reproduction, the network environment can realize the storage and transmission of multispectral images and related parameters. At the spectral reproduction end, the computer performs operations such as observational ambient light processing, spectral image processing, and spectral color correction to prepare the data to be the output for the spectral output device. In addition to this, the spectral output device is used to reproduce the spectral image, giving an image reproduction that meets the application requirements. The reproduced image can be either a spectrally matched reproduction or a color reproduction that is consistent in color appearance under different viewing conditions.

As can be seen from Figure 1, if only the reproduction of spectral matching is pursued, the red apple image at the source end may be reproduced as a purple apple, so a processing unit for color appearance matching needs to be added in the reproduction process. The multispectral image color appearance reproduction process is shown in Figure 2, and each functional module in the figure is discussed in the following sections.

The image output by the multichannel digital camera integrates various types of information such as the ambient illumination of the scene, the spectral reflection characteristics of the scene, the spectral sensitivity of the camera, and the spectral transmittance of the camera filter. To obtain reflectance data that only reflects the spectral reflection characteristics of the scene, it is necessary to use mathematical methods to estimate based on the multichannel images output by the camera, as well as the scene illumination information and the spectral characteristics of the camera. This process is called spectral reflectance reconstruction.

The process of shooting a scene by a spectral imaging system and outputting a multichannel image related to the color space of the camera can be expressed as [17]

(1) $$\begin{array}{c} d_{k}=\int_{\lambda_{\min}}^{\lambda_{\max}}s\left(\lambda \right)l\left(\lambda \right)\tau_{k}\left(\lambda \right)r\left(\lambda \right)\text{d}\lambda . \end{array}$$

Among them, *k* represents the channel, *d*_*k*_ represents the output image of the *k*th channel of the system, and *s*(*λ*) represents the spectral sensitivity of the camera. *l*(*λ*) represents the spectral power distribution of illumination, *τ*_*k*_(*λ*) represents the spectral transmittance of each channel filter, and *r*(*λ*) represents the spectral reflectance of the scene. Since spectral sensitivity, illumination spectral power distribution, and filter spectral transmittance are all sampled in the visible wavelength range, formula (1) can also be represented by the following discrete matrix:

(2) $$\begin{array}{c} D={\left(ST\right)}^{T}LR. \end{array}$$

Among them, *D* is the multichannel image output by the camera, *R* is the spectral reflectance of the scene, S is the spectral sensitivity of the camera, *L* is the spectral power distribution of the illumination, *T* is the spectral transmittance of the filter, and Θ=((**ST**)^*T*^**L**)^*T*^. We can get [18]

(3) $$\begin{array}{c} D=\Theta^{T}R. \end{array}$$

Formulas (2) and (3) are called forward models of the spectral imaging system.

The spectral reflectance reconstruction is to estimate the spectral reflectance of the scene when the abovementioned relevant characteristics and the multichannel image output by the camera are known, that is, to obtain the inverse process of the model, that is, the inverse transformation *Q*, so that

(4) $$\begin{array}{c} R=Q\;D. \end{array}$$

The learning-based reconstruction method does not require the spectral feature matrix of the imaging system in the reconstruction process. It first establishes a set of training samples (**D**, **R**) to generate the multichannel value and spectral reflectance transformation **R**_*v*_ output by the system, and

(5) $$\begin{array}{c} R_{v}=QD_{v}. \end{array}$$

*R*-matrix method situation. Among them, the *R*-matrix method takes into account the spectral information and chromaticity information contained in the device-related image in the algorithm, so it can bring better spectral reconstruction results than other methods.

The color space value of the identification system is *c*, and after identification, the spectral reflectance space value measured with the spectrophotometer is *s*; then [19],

(6) $$\begin{array}{c} s=F_{\text{print}}\left(c\right),\\ c\in \Omega_{\text{print}},\\ s\in \Omega_{\text{spec}}. \end{array}$$

Here, **F**_print_(•) represents the nonlinear mapping relationship from the recognition system color space to the spectral space, Ω_print_ represents the recognition system color space, and Ω_spec_ represents the spectral reflectance space. Correspondingly, for the spectral reflectance value that can be reproduced by the identification system, it can be transformed into the color space value of the identification system by **F**_pint_^−1^(•), namely,

(7) $$\begin{array}{c} c=F_{\text{pint}}^{-1}\left(s\right),\;s\in G_{\text{print}}. \end{array}$$

**G**_print_ represents the range of spectral values that the recognition system can reproduce, that is, the spectral domain of the recognition system. It is defined as follows:

(8) $$\begin{array}{c} G_{\text{print}}=\left\{s\in \Omega_{\text{spcc}}|\exists c\in \Omega_{\text{print}},F_{\text{print}}\left(c\right)=s\right\}. \end{array}$$

In essence, the spectral color correction of the recognition system is to obtain the forward mapping relationship **F**_print_(•) and the reverse mapping relationship **F**_pint_^−1^(•) and realize the correction transformation from the recognition system color space to the spectral space and from the spectral space to the recognition system color space. There are two main ways to find the forward and inverse transformations **F**_print_(•) and **F**_pint_^−1^(•). One is to establish an analytical mathematical recognition model, and the other is to use the lookup table method.

Color appearance matching needs to be implemented in chromaticity space, so its process can be shown in Figure 3. First, the source multispectral image is converted from the spectral color space *S*(*λ*) to the CIE chromaticity space (CIEXYZ space). Since the CIE chromaticity space can only be strictly applied to the same observation conditions of the source and the destination and it is still an observation condition dependent space, it is necessary to transform the color appearance according to the source observation conditions and convert it to the observation condition-independent space Jab_*ucs*_. Then, according to the reproduction and observation conditions, the color appearance inverse transformation is performed to obtain the chromaticity value *X*′*Y*′*Z*′ with the same color appearance under the reproduction and observation conditions, and finally, the chromaticity inversion is performed to obtain the reproduction spectral reflectance image *S*′(*λ*).

The chromaticity transformation only needs to integrate the source multispectral image data, illumination information, and the color vision characteristics of the observer. The method of color appearance transformation will not be repeated here. The process of chrominance inversion is more complicated than chrominance transformation, which includes high-dimensional spectral estimation and spectral modulation.

*T* represents the chromaticity value obtained after the color appearance is reversed, and *s* represents the spectral reflectance estimated from the tristimulus value *t*; then, the relationship between *t* and *s* can be expressed as

(9) $$\begin{array}{c} t={\left[\begin{array}{ccc} X & Y & Z \end{array}\right]}^{T}=kFLs. \end{array}$$

Here, $F={\left[\begin{array}{ccc} \bar{x}\left(\lambda \right) & \bar{y}\left(\lambda \right) & \bar{z}\left(\lambda \right) \end{array}\right]}^{T}$ represents the standard observer color matching function, and **L**=diag(**l**(*λ*)) represents a diagonal matrix with the spectral power distribution **l**(*λ*) of the reproduced illumination as the diagonal elements.

We set

(10) $$\begin{array}{c} {\left[\begin{array}{ccc} X_{\text{illum}} & Y_{\text{illum}} & Z_{\text{illum}} \end{array}\right]}^{T}=F\cdot L\cdot \text{ones}\left(1\right). \end{array}$$

Here, ones (1) represents an all-ones vector. To make the *Y* value of white light 100, we set

(11) $$\begin{array}{c} k=\frac{100}{Y_{\text{illum}}}, \end{array}$$

*c* is the tristimulus value normalized to the [0, 1] interval of each component, namely,

(12) $$\begin{array}{c} c={\left[\begin{array}{ccc} X_{\text{Norm}} & Y_{\text{Norm}} & Z_{\text{Norm}} \end{array}\right]}^{T}={\left[\begin{array}{ccc} \frac{X}{X_{N}} & \frac{Y}{Y_{N}} & \frac{Z}{Z_{N}} \end{array}\right]}^{T}, \end{array}$$

(13) $$\begin{array}{c} {\left[\begin{array}{ccc} X_{N} & Y_{N} & Z_{N} \end{array}\right]}^{T}=k\cdot F\cdot L\cdot \left(1\right). \end{array}$$

Through formulas (9) to (13), the transformation between the spectral reflectance *s* can be estimated and the normalized tristimulus value *c* can be established [20]:

(14) $$\begin{array}{c} c=Ds\;. \end{array}$$

Here,

(15) $$\begin{array}{c} D=\text{NFL,}\\ N=\text{diag}\left({\left[\begin{array}{ccc} \frac{k}{X_{N}} & \frac{k}{Y_{N}} & \frac{k}{Z_{N}} \end{array}\right]}^{T}\right)=\text{diag}\left({\left[\begin{array}{ccc} \frac{1}{X_{\text{illum}}} & \frac{1}{Y_{\text{illum}}} & \frac{1}{Z_{\text{illum}}} \end{array}\right]}^{T}\right). \end{array}$$

For a set of *n* spectral reflectance **S** , formula (14) can be generalized as

(16) $$\begin{array}{c} C=DS. \end{array}$$

Here, $C=\left[\begin{array}{cccc} c_{1} & c_{2} & \cdots & c_{n} \end{array}\right]\text{ and}\;S=\left[\begin{array}{cccc} s_{1} & s_{2} & \cdots & s_{n} \end{array}\right].$

This section needs to solve the inverse problem of (14), that is, to estimate the spectral reflectance *s* from the normalized tristimulus value *c*, and *H* is the estimation matrix; then, the high-dimensional spectral estimation formula is

(17) $$\begin{array}{c} s=Hc. \end{array}$$

For the chrominance image after color appearance inversion, it can be generalized as

(18) $$\begin{array}{c} S=HC. \end{array}$$

To calculate the matrix *H*, first, we select a set of samples with known spectral reflectance (this paper selects the standard target IT8.7/3 as the sample set, and the number of samples is 928), denoted as $\bar{S}$. According to formula (16), the normalized tristimulus value set of the sample set under the reproduction observation environment can be obtained, namely,

(19) $$\begin{array}{c} \bar{C}=D\bar{S}. \end{array}$$

Second, the transformation from the normalized tristimulus value set to the spectral reflectance sample set can be established by estimating the matrix *H*:

(20) $$\begin{array}{c} \bar{S}=H\bar{C}. \end{array}$$

It can be seen from the previous formula that *H* is the generalized inverse matrix of matrix *D*, which can be obtained by calculating $\bar{S}$ and $\bar{C}$. Multiplying both sides of formula (20) by ${\bar{C}}^{T}{\left(\bar{C}{\bar{C}}^{T}\right)}^{-1}$, we have

(21) $$\begin{array}{c} \bar{S}{\bar{C}}^{T}{\left({\bar{CC}}^{T}\right)}^{-1}=H{\bar{CC}}^{T}{\left(\bar{C}{\bar{C}}^{T}\right)}^{-1}. \end{array}$$

From this, it can be obtained [21]:

(22) $$\begin{array}{c} H=\bar{S}{\bar{C}}^{T}{\left(\bar{C}{\bar{C}}^{T}\right)}^{-1}. \end{array}$$

After calculating the matrix *H* and substituting it into formula (18), the high-dimensional spectrum S can be estimated from the chromaticity space image after the color appearance inversion.

Due to the existence of metamerism, there should be an infinite number of spectral reflectances corresponding to a tristimulus value. In formula (18), H is the generalized inverse matrix of *D*, which determines that the spectral reflectance *s* estimated by the normalized tristimulus value *c* through (18) is only one of the infinite metamerism colors that reproduce the observation environment. It achieves color appearance matching with the source image spectrum $\hat{S}$ before chroma transformation, but there is a large spectral error. Since both spectral matching and color appearance matching are critical to the reproduction quality of an image, in order to achieve (or approximate) spectral matching with the source spectral data, it is necessary to correct the estimated spectrum *s* to obtain the final reproduced spectrum *S*′. The metamerism of *S*′ and *S* under the condition of reproduction observation, but the spectral error with the source spectrum $\hat{S}$ is smaller; this process is called spectral modulation, denoted as

(23) $$\begin{array}{c} S{}^{\prime }=\text{MC}\left(\hat{S},S\right). \end{array}$$

Here, MC(·) represents the spectral modulation function.

In order to realize the spectral modulation function, the estimated spectrum can be decomposed by R-matrix theory. The matrix is essentially an orthogonal projection operator, which is defined as

(24) $$\begin{array}{c} R=A{\left(A^{T}A\right)}^{-1}A^{T}. \end{array}$$

Here, *A* is the combined action matrix of the reproduced illumination spectrum and the standard observer, which can be expressed as

(25) $$\begin{array}{c} A=k\cdot L\cdot F. \end{array}$$

The fundamental stimulus **S**^*∗*^ of the spectrum S is the projection of *S* on *R*, that is,

(26) $$\begin{array}{c} S^{*}=RS,\\ B=\left(I-R\right)\hat{S}. \end{array}$$

Here, **I** represents the identity matrix. Therefore, the final reproduced spectrum should be

(27) $$\begin{array}{c} S^{\prime }=S^{*}+B. \end{array}$$

CMM is the core of color processing, and the working principle of spectral color appearance reproduction CMM is shown in Figure 4.

For any spectral image acquired by the spectral imaging system, the CMM uses the observed ambient illumination provided in the source spectrum profile and the characteristic parameters of the spectral imaging system to reconstruct the spectral reflectance to obtain the spectral reflectance vector value of each pixel of the spectral image. Then, it uses the observation condition information provided in the source and destination profiles to perform color appearance matching and to obtain a spectrally approximated reproduced spectral reflectance image that matches the color appearance of the source spectral reflectance image. When the image is reproduced, according to the characteristic parameters of the output device provided in the target spectrum profile, the reproduced spectral reflectance data is transformed into the color space of the output device and then the reproduced image is obtained through the output device.

As can be seen from Figure 4, the spectral color appearance reproduction CMM mainly includes three independent real-time calculation modules: spectral reflectance reconstruction, color appearance matching, and spectral color correction. Among them, the spectral reflectance reconstruction method has a relatively mature algorithm at present, and the experiment proves that the R-matrix method based on learning can obtain higher reconstruction accuracy. Spectral color correction can use two methods given in the literature: color correction method based on identifying spectral model and color correction method based on lookup table. When performing color appearance matching, the CMM first reads out the image from the source spectrum profile to obtain the illumination information of the environment and obtains the chromaticity value of the source spectrum image. Then, it reads out the source and destination observation condition information from the source profile and the destination profile, respectively, and performs color appearance transformation and inversion. After that, it calculates the estimation matrix H according to the spectral reflectance sample set and reestimates the high-dimensional spectrum. Finally, it uses the source reconstructed spectral reflectance data as a standard to spectrally modulate the estimated spectrum to obtain the reconstructed spectral reflectance. The process of color appearance matching performed by the CMM is shown in Figure 5.

## 4. Evaluation of Physical Education Teaching Effect Based on Action Skill Recognition

The flow of the physical education effect evaluation system based on action skill recognition is shown in Figure 6.

In this process, the initial camera parameter calculation module adopts a method basically similar to the court. Since the camera of the court is in a nonfixed state, the camera parameters need to be calculated in real time, which makes it necessary to consider the system overhead caused by the perspective transformation matrix calculation in addition to video fusion and moving object segmentation. In order to meet the real-time requirements, we designed a method using feature point estimation and direct line fitting according to the distribution characteristics of feature points in consecutive video frames.  Figure 7 shows the digitized image for action recognition.

This paper analyzes the physical education effect evaluation system based on action skill recognition proposed in this paper through multiple sets of experiments and counts the accuracy rate of movement recognition and physical education teaching effect of this system. The test results shown in Table 1 are obtained.

The above test results verify that the physical education effect evaluation system based on action skill recognition meets the actual needs of physical education and has a good role in promoting the recognition of physical skills and the improvement of physical education effects.

## 5. Conclusion

Physical education is one of the basic teaching organization forms in school education, and it is an important path for cultivating talents with comprehensive development of morality, intelligence, physique, and beauty. Moreover, physical education is a bilateral teaching activity that teachers and students participate in and cooperate with each other under the guidance of physical education teachers. The quality of physical education teaching is directly related to the physical and mental health of students and also related to the professional growth and development of teachers. It is an important educational practice link in the school education system. Both the implementers and participants in teaching activities are driven by the power of teaching and promote the development of physical education. This paper combines the action skill recognition algorithm to construct the physical education teaching effect evaluation system. The simulation experiment verifies that the physical education effect evaluation system based on action skill recognition meets the actual needs of physical education and has a good role in promoting the recognition of physical skills and the improvement of physical education effect.

## Figures and Tables

**Figure 1:** Schematic diagram of the multispectral image reproduction process.

**Figure 2:** Flow chart of color appearance reproduction in multispectral images.

**Figure 3:** Flow chart of color appearance matching.

**Figure 4:** Basic working principle of spectral color appearance reproduction CMM.

**Figure 5:** Schematic diagram of color appearance matching process.

**Figure 6:** Flow of the physical education teaching effect evaluation system based on motor skill recognition.

**Figure 7:** An example of a digitized image for motion recognition. (a) Original image of sports action. (b) Background removal of sports action. (c) Feature recognition of sports actions.

**Table 1:** Effect verification of the physical education teaching effect evaluation system based on motor skill recognition.

Number	Action recognition	Teaching effect	Number	Action recognition	Teaching effect
1	89.28	81.42	23	93.99	80.22
2	88.80	87.64	24	90.85	85.55
3	88.67	87.11	25	92.47	83.98
4	91.24	84.05	26	89.52	82.96
5	92.20	78.84	27	90.84	84.35
6	93.49	85.10	28	87.96	88.87
7	90.63	80.45	29	91.31	88.64
8	89.23	88.26	30	93.29	78.84
9	88.65	84.45	31	88.46	80.48
10	90.46	82.54	32	87.92	81.58
11	91.64	81.49	33	87.55	82.70
12	92.60	85.49	34	93.44	83.83
13	93.11	85.07	35	93.89	78.29
14	92.49	88.52	36	92.83	80.31
15	87.23	80.40	37	89.14	78.43
16	91.22	88.65	38	90.81	85.35
17	89.44	85.08	39	88.06	84.53
18	89.66	82.77	40	87.14	88.07
19	87.87	79.36	41	87.27	88.11
20	92.68	85.00	42	88.24	84.29
21	91.73	86.66	43	89.65	82.91
22	92.52	88.09	44	87.31	85.42

## Data Availability

The labeled dataset used to support the findings of this study are available from the corresponding author upon request.
